# Clinical predictors of incident gallstone disease in a Chinese population in Taipei, Taiwan

**DOI:** 10.1186/1471-230X-14-83

**Published:** 2014-04-28

**Authors:** Jau-Yuan Chen, Chung-Te Hsu, Jorn-Hon Liu, Tao-Hsin Tung

**Affiliations:** 1 Department of Family Medicine, Linkou Chang-Gung Memorial Hospital and Chang-Gung University, Taoyuan, Taiwan; 2 Cheng Hsin General Hospital, Taipei, Taiwan; 3 Cheng Hsin General Hospital; Faculty of Medicine, School of Medicine, National Yang-Ming University, Taipei, Taiwan; 4 Cheng Hsin General Hospital; Faculty of Public Health, School of Medicine, Fu-Jen Catholic University, Taipei, Taiwan

**Keywords:** Follow-up study, Gallstone disease (GSD), Incidence density, Predictive factors, Screening

## Abstract

**Background:**

Gallstone disease (GSD) is a common gastrointestinal disorder throughout the world. The authors explored the incidence of GSD in Taiwan and its condition-associated predictive factors.

**Methods:**

The initial study cohort comprised 2386 healthy adult participants, who were voluntarily admitted to a teaching hospital for a physical check-up in 2002 in Taipei, Taiwan. After excluding 126 patients who exhibited prevalent GSD, 2260 non-GSD participants received annual follow-up screenings for GSD until 31 December, 2007. Of those, 1296 (57.3%) patients were re-examined to collect blood samples and conduct ultrasound sonography.

**Results:**

Among the 1296 participants who exhibited no GSD at the first screening, 23 patients developed GSD during 3640 person-years of follow-up. The incidence was 0.632% per year (95% CI: 0.292%–2.009%). After conducting a Cox regression, increased age (50–59 years versus < 40 years, RR = 2.16 [95% CI: 1.09–5.97], 60+ years versus < 40 years, RR = 3.81 [95% CI: 2.77–8.63]), high body mass index (≥27 kg/m^2^ versus < 24 kg/m^2^, RR = 1.64 [95% CI: 1.07–2.98]), high fasting plasma glucose levels (≥126 mg/dL versus < 110 mg/dL, RR = 1.68, 95% CI: 1.10–3.87), and nonalcoholic fatty liver disease (yes versus no, RR = 1.44, 95% CI: 1.21–1.90) appeared to be significantly related to developing GSD.

**Conclusion:**

Increased age is a well-established risk factor for developing GSD. The current findings indicated that high body mass index, elevated fasting plasma glucose levels, and nonalcoholic fatty liver disease were also associated with GSD.

## Background

Gallstone disease (GSD), a digestive disorder with multifactorial origins, is a common gastrointestinal disorder throughout the world. The third National Health and Nutrition Examination Survey estimated that 6.3 million men and 14.2 million women ages 20–74 in the United States had GSD [1]. Although GSD yields a low mortality rate, an increased risk of overall mortality in GSD patients is not entirely explained by the high rate of associated cancer deaths; thus, this high morbidity substantially affects the economy and public health [2]. Because of the Westernization of the Taiwanese diet and environment, GSD is no longer rare among its Chinese population and has become a major health problem [3]. In the absence of a suitable screening program for symptomatic GSD, treating GSD and related complications yields substantial healthcare costs.

The availability of ultrasonography as an accurate tool for GSD diagnosis has facilitated evaluating GSD morbidity by conducting epidemiological surveys of the general population [2,4,5]. Previous research has explored the prevalence of GSD and its associated factors [3]. Although cross-sectional studies provide useful information regarding disease prevalence, they fail to address the incidence or new cases of GSD among the study population. Thus, the population must be re-examined after a period of time to determine the incidence and causal relations between the risk factors and disease. From a preventive medicine perspective, GSD prevention should focus the relevant risk factors of the disease; thus, exploring the incidence and risk factors of GSD is essential for preventing its development and the cholecystectomy caused complications, which are often insidious. Therefore, a cohort study was indicated for estimating the incidence of GSD; we explored the incidence and risk factors of GSD in Taipei, Taiwan, using a 5-year follow-up period and real-time abdominal ultrasound data.

## Methods

### Data resource and data collection

Figure 1 shows the procedures for GSD screening between 2002 and 2007. We first established a study cohort to determine the incidence of GSD; the initial study cohort comprised 2386 healthy adults (1235 males and 1151 females) who were voluntarily admitted to a teaching hospital for a physical check-up between January 2002 and December 2002 in Northern Taiwan. Of the 2386 patients, 126 were diagnosed with GSD. The overall prevalence of GSD was 5.3%, comprising single stone 1.7% (n = 40), multiple stone 2.3% (n = 55), and cholecystectomy 1.3% (n = 31) [3]. The details of the study design and execution have been described in full elsewhere [3]. Subsequent annual follow-up screenings for GSD were conducted until 31 December, 2007 for the 2260 patients invited by telephone calls or invitation letters in receive general health examinations and abdominal examinations who lacked GSD in 2002. Participants who were diagnosed as GSD or known cholecystectomy for GSD at the first screening were separately studied [6].

**Figure 1:** The procedure of screening for gallstone disease among healthy adults during 2002–2007.

We analyzed all patients who participated in at least two GSD screenings, but 964 (42.7%) failed to complete the series of assessments. Those who lost to follow-up during the 5-year period were older (50.9 ± 10.2 years versus 45.1 ± 9.5 years, *P* < .0001), and exhibited higher systolic blood pressure (SBP) levels (126.2 ± 20.4 mmHg versus 119.0 ± 16.7 mmHg, *P* < .0001) and fasting plasma glucose (FPG) levels (103.8 ± 23.0 mg/dL versus 95.7 ± 24.6 mg/dL, *P* < .0001) compared with the participants. All procedures were performed in accordance with the guidelines of the relevant institutional ethics committee, adhering to the Declaration of Helsinki. The participant information was anonymous and taken from the hospital database. This access to personal records was approved to use blood samples and ultrasound sonography results and that these were collected as part of standard care by the human subject review board of Cheng-Hsin General Hospital (CHGH-IRB: (137)97-26) in Taipei, Taiwan.

Blood samples were collected and ultrasound sonography was conducted. Clinical nurses drew fasting blood samples from the study participants by using venipuncture. Overnight-fasting serum and plasma samples (from whole blood preserved using EDTA and NaF) were maintained frozen at −20°C until analysis. We defined type-2 diabetes (FPG ≥ 126 mg/dL) based on the 1997 ADA criteria [7], using the following conditions: obesity as a body mass index (BMI) ≥ 27 kg/m [2], high SBP ≥ 140 mmHg, high diastolic blood pressure ≥ 90 mmHg, hypercholesterolemia (≥200 mg/dL), hypertriglyceridemia (≥200 mg/dL), low HDL (<35 mg/dL), high blood urea nitrogen (BUN; ≥ 20 mg/dL), high creatinine (≥1.4 mg/dL), and hyperuricemia (≥7 mg/dL for males or ≥ 6 mg/dL for females). Serum alanine transaminase (ALT) or aspartate transaminase (AST) levels of ≥ 40 U/L were classified as elevated [8]. In addition, the related demographic information, dietary habits, and other personal and family chronic diseases history were collected at one-to-one well-trained interviews using a structured questionnaire.

### Diagnosis of gallstone disease and nonalcoholic fatty liver disease

After at least 8 hours of fasting, a panel of specialists examined the abdominal region of each patient, diagnosing GSD based on real-time ultrasound sonography (TOSHIBA nemio SSA-550A, Japan) and the presence of “movable hyper-echoic foci with acoustic shadows.” Cases of GSD were classified as follows: single gallbladder stone, multiple gallbladder stones, and cholecystectomy, excluding gallbladder polyps. The cases were identified as any type of GSD that developed among the study population [3].

The ultrasonographic criteria which were used to diagnose a fatty liver included liver and kidney echo discrepancy, presence of an increased liver echogenicity, echo penetration into the deep portion of the liver, and clarity of the liver blood vessel structures [9]. All study subjects who were diagnosed as nonalcoholic fatty liver disease (NAFLD) by ultrasound and without disease history of Wilson’s disease, intestinal bypass surgery, or gulten enteropathy, ingestion of of drugs known to produce hepaticsteatosis including methotrexate, tamoxifen, amiodarone, and nucleoside analogues, positive serology for hepatitis B or C virus, a history of another known liver disease, and alcohol consumption (alcohol intake of 30 g/day or more for males and 20 g/day or more for females) were enrolled the study [10].

### Interobserver reliability in ultrasound sonography

To establish a consistent GSD diagnoses among the specialists, we used the Kappa statistic to assess the agreement of interobserver reliability. We conducted a pilot study, randomly selecting 100 non-study participants. Regarding interobserver reliability, the Kappa value for GSD diagnosis among specialists was 0.79 (95% CI: 0.61–0.95) [3]. In addition, the Kappa value for diagnosis of NAFLD between specialists was 0.77 (95% CI: 0.69-0.88).

### Statistical analysis

We performed statistical analyses using SAS for Windows, (SAS version 9.0; SAS Institute Inc., Cary, NC, USA), determining the GSD incidence per year based on the ratio of the observed number of cases to the total number of patient-years at risk. The 95% confidence intervals (95% CI) were calculated for incidence by using a Poisson distribution. Concerning the univariate analysis, a *t*-test and chi-square test were used to evaluate the continuous and categorical variables; a multiple Cox regression was conducted to investigate the independence of factors associated with developing GSD. A *P* value of < 0.05 was considered statistically significant. The results are presented as mean ± SD.

## Results

Of the 2260 participants in the study cohort, 1296 attended at least 2 sonographic check-ups: 710 (54.8%) attended 2 consultations, 402 (31.0%) attended 3 consultations, and 184 (14.2%) attended 4 or more consultations during the 5-year period. The overall response rate was approximately 57.3, and the mean follow-up time was 3.51 ± 0.84 years. The patients were considered censored cases if their outcomes were unavailable. Twenty participants were found to have GSD (9 single stone and 11 multiple stones) and three had received cholecystectomy for GSD during the 5-year follow-up period. Table 1 shows that the females attained higher attendance rates than the males did (62.3% versus 52.8%) and young people (<40 and 40–49 years) exhibited a slightly lower attendance rate compared with other age groups.

**Table 1:** The attendance rate of gallstone disease screening from 2002 to 2007 (n = 1296)

**Variable**	**Eligible population**	**Screened population**	**Attendance rate**
	***n***	***n***	**(%)**
**Sex**			
Male	1176	621	52.8
Female	1084	675	62.3
**Age**			
<40	734	373	50.8
40-49	704	409	58.1
50-59	464	285	61.4
60+	358	229	64.0
**Total**	2260	1296	57.3

Table 2 lists the gender- and age-specific incidences of GSD. The overall incidence of GSD was 0.632% per year (95% CI: 0.292%–2.009%), indicating a clear trend based on age (p = 0.03), where values monotonically increase. The values increased from 0.214% per year (95% CI: 0.062%–1.719%) at ages <40 to 0.470% per year (95% CI: 0.112%–2.103) at ages 40–49, 0.585% per year (95% CI: 0.236%–1.983%) at ages 50–59, and 1.394% per year (95% CI: 0.410–2.477%) at ages greater than 60. The age groups exhibited no consistent patterns. Females demonstrated a slightly higher incidence (0.741% versus 0.496% per year, *P* = 0.40) compared with males, but the gender difference was non-significant.

**Table 2:** Sex- and age-specific incidence of gallstone disease among screened patients (n = 1296)

**Incidence of any gallstone disease**				
**Variable**	**No. of no GSD at first screening**	**New cases**	**Person years at risk**	**Incidence Density (% per year) (95% CI)**
**Gender**				
Male	621	8	1614.5	0.496 (0.181-1.973)
Female	675	15	2025.5	0.741 (0.254-2.116)
p-value				0.40
**Age**				
<40	373	2	932.5	0.214 (0.062-1.719)
40-49	409	5	1063.5	0.470 (0.112-2.103)
50-59	285	5	855	0.585 (0.236-1.983)
60+	229	11	789	1.394 (0.410-2.477)
p-value				0.03
Total	1296	23	3640	0.632 (0.292-2.009)

Table 3 shows the risk factors for developing GSD based on the univariate analysis. The significant risk factors of GSD were age (*P* < .0001), FPG (*P* < .0001), SBP (*P* < .0001), BMI (*P* < .0001), ALT (*P* = .001), and NAFLD (*P* = .04). In addition, to assess how these factors independently contributed to GSD, the significant variables from the univariate analysis were examined using a Cox regression, evaluating age, FPG, SBP, BMI, ALT, and NAFLD. As Table 4 shows, subsequent to adjustment for confounders, the following factors appeared to be significantly related to GSD incidence: age (50–59 years versus < 40 years, RR = 2.16 [95% CI: 1.09–5.97], 60+ years versus < 40 years, RR = 3.81 [95% CI: 2.77–8.63]), elevated BMI (≥27 kg/m^2^ versus < 24 kg/m^2^, RR = 1.64 [95% CI: 1.07–2.98]), elevated FPG (≥126 mg/ dL versus <110 mg/dL, RR = 1.68, 95% CI: 1.10–3.87), and NAFLD(yes versus no, RR = 1.44, 95% CI: 1.21–1.90).

**Table 3:** Univariate analysis of risk factors for the development of gallstone disease among screened patients (n = 1296)

		**Development of gallstone disease**			
**Variables**		**Yes (n = 23)**	**No (n = 1273)**	**P value for t test or chi-square test**	**Definitions of disease condition**
		**Mean ± SD**	**Mean ± SD**		
**Continuous variables**					
Age (years)		60.55 ± 14.28	51.32 ± 13.01	<0.0001	----
Fasting plasma glucose (mg/dL)		113.78 ± 20.69	100.55 ± 30.06	<0.0001	≥126 mg/dL
Systolic blood pressure (mmHg)		132.90 ± 19.77	123.08 ± 18.69	<0.0001	≥140 mmHg
Diastolic blood pressure (mmHg)		80.77 ± 11.90	79.23 ± 12.07	NS	≥90 mmHg
Body mass index (Kg/m^2^)		24.86 ± 3.48	23.39 ± 3.37	<0.0001	≥27Kg/m^2^
Total cholesterol (mg/dL)		218.17 ± 35.68	209.80 ± 36.75	NS	≥200 mg/dL
Triglyceride (mg/dL)		150.68 ± 88.04	147.26 ± 79.53	NS	≥200 mg/dL
HDL (mg/dL)		55.70 ± 16.31	54.24 ± 15.92	NS	<35 mg/dL
BUN (mg/dL)		14.82 ± 6.19	14.57 ± 5.80	NS	≥20 mg/dL
Creatinine (mg/dL)		1.07 ± 0.33	1.05 ± 0.28	NS	≥1.4 mg/dL
AST (U/L)		30.78 ± 19.61	27.08 ± 18.55	NS	≥40U/L
ALT (U/L)		34.42 ± 22.06	28.19 ± 21.50	0.001	≥40U/L
Uric acid (mg/dL)		6.05 ± 1.01	5.99 ± 1.12	NS	≥7 mg/dL for males or ≥6 mg/dL for females
**Categorical variables**					
NAFLD	yes	17 (73.9%)	672 (52.8%)	0.04	----
	no	6 (26.1%)	601 (47.2%)		----
Heavy fatty or fried foods	yes	5 (21.7%)	251 (19.7%)	NS	----
	no	18 (78.3%)	1022 (80.3%)		----

**Table 4:** Cox regression model of risk factors associated with the development of gallstone disease among screened patients (n = 1296)

	**Development of gallstone disease (yes versus no)**	
**Variables**	**Relative risk**	**(95% CI)**
Gender (female versus male)	2.12	0.45-4.16
Age (40–49 versus <40 years)	1.65	0.41-3.79
(50–59 versus <40 years)	2.16	1.09-5.97
(60+ versus <40 years)	3.81	2.77-8.63
BMI (24–27 versus <24 Kg/m^2^)	1.13	0.56-3.28
(≥27 versus <24 Kg/m^2^)	1.64	1.07-2.98
FPG (110–125 versus <110 mg/dL)	1.22	0.49-2.31
(≥126 versus <110 mg/dL)	1.68	1.10-3.87
Higher SBP (yes versus no)	1.11	0.53-2.18
Higher ALT (yes versus no)	1.03	0.68-2.87
NAFLD (yes versus no)	1.44	1.21-1.90

## Discussion

### Incidence and risk factors for the development of gallstone disease

Knowledge of GSD epidemiology is crucial to managing this disorder when planning preventive programs and identifying the optimal therapeutic strategies [2]. Previous clinical studies have yielded reliable positive (0.99–1.00) and negative (0.90–0.96) predictive values regarding the diagnostic efficacy of ultrasonography [11], suggesting that abdominal ultrasound is a robust method for GSD screening. The availability of ultrasonography as an accurate tool for GSD diagnosis has facilitated evaluating GSD morbidity by conducting epidemiological surveys of study populations in Eastern and Western countries [2,3,12,13]. Few studies have explored the incidence and possible etiology of GSD among the general population of Taiwan.

The incidence of GSD appears to vary among test populations and differs among studies conducted in disparate countries [2,12,13]. It is of interest that the prevalence and the incidence differ very little from two Italian studies, 10 years apart - GREPCO (1998) and MICOL (2008) [2,13]. This may suggest that the diet of the Chinese in Taiwan is already Westernised. In addition to varying methods of assessing GSD, this disparity might be caused by differences among genetic populations. In this study, the annual incidence of overall GSD was slightly lower compared with that of other evidence-based studies [2,13]; this difference may be a result of the Kappa value for the agreement of interobserver reliability. Although the value appeared appropriate [14], non-differential misclassification-bias identification could have occurred, generating an underestimated GSD incidence.

In this study, the proportion of the population lost to follow up was in the higher risk categories for GSD. This deficiency is likely to have under recorded the overall incidence. In addition, the response rate was lower than that reported in other follow-up studies for GSD [2,12,13] and the older population had a higher attendance rate could be related a potential self-selection bias. The characteristics of the elderly subjects which may cause them to select themselves in the screening program create abnormal or undesirable conditions in the group.

The estimated incidence of GSD in this study was higher in females compared with males, and increased as age increased. This finding is consistent with the reports of other studies conducted elsewhere [2,13]. GSD is rare in neonates and young children [5]; thus, long-term exposure to risk factors may explain the increased probability of developing GSD in old age. The morbidity of GSD increases as age increases, noticeably elevating after age 40 and becoming 4- to 10-fold more likely [15]. Although GSD patients are often clinically silent, the symptoms of GSD and number of severe complications increase as age increases, leading to cholecystectomy in more than 40% of patients older than 40 [5,16]. In addition, gender is a substantial factor in GSD and females are almost twice as likely as males to develop stones [15]. Female sex hormones adversely influence hepatic bile secretion and gallbladder function and estrogens increase cholesterol secretion and diminish bile salt secretion [5]. Thus, females do not have a significantly higher incidence of all types of GSD compared with males. Another possible reason was that a Type II error due to small incident numbers, since the relative risk is 2.12 in this study. Previous research has shown that cholesterol GSD is common among Western populations, whereas pigment GSD is common in Taiwan [17]. The differing findings among Eastern and Western populations suggests that cholesterol GSD is not yet a major problem among Chinese populations.

The findings indicated that FPG ≥ 126 mg/dL was highly associated with GSD incidence; that is, type 2 diabetes might be a positive risk factor for GSD. The association between diabetes mellitus and GSD is confounded by age, obesity, and family history of GSD [15]. The possible pathogenic reasons for this are that type 2 diabetes combined with GSD might induce acute cholecystitis more often and yield a higher probability of progression to septicemia compared with non-diabetic patients, who exhibit normally functioning gallbladders. Late-onset diabetes patients may demonstrate a higher lithogenic bile index compared with non-diabetics after adjusting for sex and age [18]. The association between diabetes and GSD is stronger among patients who have a history of treated diabetes mellitus than it is among those with a simple history of diabetes; this could indicate that hyperglycemia affects gallbladder motility [3]. In addition, the links among diabetes, obesity, and GSD most likely originate from metabolic syndrome [15,19].

After using univariate and multiple Cox regression analyses, the findings indicate that obesity is a significant risk factor for GSD. This agreed with the results of other studies that employed extended screening intervals [2,12,13]. The validity of BMI as a measure of adiposity has been assessed by comparison with densitometry [12]. From a biological viewpoint, BMI is primarily a surrogate of lean body mass when BMI and height-adjusted waist circumference are included in the same model, because the variation in BMI attributable to adiposity is essentially controlled by the height-adjusted waist circumference variable [12,18]. However, additional epidemiological and etiologic investigations must explore the pathophysiological mechanisms among BMI, waist circumference, and GSD among Chinese populations.

Cirrhosis is a predictive risk factor for GSD, particularly in the advanced stages of the disease [20,21]. The annual incidence of GSD among cirrhosis patients is approximately 8 times higher than is that among the general population [20]. ALT has, for some time, been viewed as a sensitive indicator of liver-cell injury [22]. Determining serum ALT levels is the most frequent test used to identify liver disease. This parameter also acts as a surrogate marker for disease severity and an index of hepatic activity [18]. In addition to type 2 diabetes, the findings show that elevated ALT levels may indicate an increased risk of GSD, implying that appropriately integrated diagnosis and therapy in the early stages of liver dysfunction might facilitate preventing GSD. Additional studies should be conducted to explore whether elevated ALT levels are an indicator of GSD, rather than a sign of serious liver diseases, such as cirrhosis, because they can indicate a fatty liver (and thus a high BMI) and the early stages of chronic liver disease [18].

NAFLD includes a wide spectrum of liver diseases, ranging from simple fatty liver, simple steatosis, nonalcoholic steatohepatitis (NASH), and liver cirrhosis, which may eventually progress to liver damage, liver fibrosis, portal hypertension, and hepatocellular carcinoma [23]. In mainland China and Taiwan, NAFLD is now viewed as one of major causes of asymptomatic elevation of liver enzymes [24,25]. Our results indicated that NAFLD was associated with incident GSD after adjustment for confounding factors.The association between NAFLD and GSD is based upon associated risk factors and metabolic derangements that are common to both conditions. From the preventive medicine viewpoint, modifiable risk factors for GSD and NAFLD include obesity and metabolic syndrome, both of which can be addressed with weight loss, exercise and dietary modifications such as a low-fat, low-sugar diet [26].

### Methodological considerations

Although we used a follow-up study design to clarify the temporal characteristics of the potential risk factors of GSD, certain limitations apply to this study. First, a major limitation was the potential self-selection bias caused by the hospital-based study design and those aged 60 or over were only 18% of the sample and yet developed 48% of the GSD; that is, the sample may not be representative of the general population. Second, the risk characteristics pertinent to the study participants significantly differed from those of non-respondents, indicating that the patients who did not complete the follow-up might have severe GSD. We assumed that all new GSD cases occurred during screening year; however, because additional GSD cases could occur at any time during the screening period, the incidence of GSD could be underestimated. Third, we did estimate the incidence of GSD formation, but rather investigated the incidence of newly screened GSD, focusing only on clinically relevant GSD. Fourth, we did not distinguish between cholesterol and pigment stones, potentially yielding measurement errors and distinct pathogenicity. Fifth, the incidence of GSD was higher (although non-significant) in female, however, there are no data regarding the number of pregnancies and the frequency of pill in this study. Finally, we further explored the 964 out of 2260 subjects who were lost to follow-up using telephone interview: 29 cases deceased, 106 cases moved out of the study township, 281 cases were refusals, 12 cases had presence of GSD or history of cholecystectomy. This might imply that the sample size was insufficient to estimate how potential risk factors affect the incidence of GSD. Further long-term research should be conducted to explore the morbidity of GSD and plausible biological mechanisms underlying its development.

## Conclusion

Increased age is a well-established risk factor for the development of GSD. The current findings indicate that high BMI, elevated FPG and NAFLD levels are also associated with GSD.

## Competing interests

The authors declare that they have no competing interests.

## Authors’ contributions

T-HT and C-TH executed the study and drafted the manuscript. J-YC and T-HT participated in the study design and performed the statistical analyses. T-HT and J-HL envisioned the study and coordinated drafting the manuscript. All authors read and approved the final version of the manuscript.

## Pre-publication history

The pre-publication history for this paper can be accessed here:

http://www.biomedcentral.com/1471-230X/14/83/prepub
